# Effects of Pulsed Radiofrequency on Nerve Repair and Expressions of GFAP and GDNF in Rats with Neuropathic Pain

**DOI:** 10.1155/2021/9916978

**Published:** 2021-09-17

**Authors:** Qing Zhu, Yi Yan, Daying Zhang, Qingtian Luo, Cuihua Jiang

**Affiliations:** ^1^Department of Pain, Ganzhou Hospital Affiliated of Nanchang University, Ganzhou, 341000 Jiangxi Province, China; ^2^Department of Pain, The First Affiliated Hospital of Nanchang University, Nanchang, 330000 Jiangxi Province, China; ^3^Department of Gastroenterology, Ganzhou Hospital Affiliated of Nanchang University, Ganzhou, 341000 Jiangxi Province, China

## Abstract

**Objective:**

To study the effect of pulsed radio frequency (PRF) on nerve repair and the expression of GFAP and GDNF in rats with neuropathic pain.

**Methods:**

Thirty SPF healthy SD rats were randomly divided into control group (Group C), PSNL group (partial ligation of sciatic nerve) + sham group (Group PS), and PSNL group (partial ligation of sciatic nerve) + PRF group (Group PR), with 10 rats in each group. In group C, the right sciatic nerve was exposed without ligation. In the PS group, the model of neuropathic pain was established by partial ligation of sciatic nerve. The mice in the PR group were treated with PRF after establishing the neuropathic pain model. The general behavior of rats during the treatment was observed. The mechanical and thermal hyperalgesia were measured before operation and 1, 3, 7, and 14 days after operation. The content of inflammatory factors in nerve tissue was detected by ELISA. The pathological condition of nerve tissue was observed by HE. The gene and protein changes of GFAP and GDNF in nerve tissue were determined by QRT PCR and Western blot.

**Results:**

Rats in the control group were free to move and in good condition. In the PS group, there were different degrees of claudication, weakness of the lower limbs, lateral toe valgus, nerve injury, and other behavioral changes. After the pulsed radiofrequency in the PR group, the above symptoms decreased gradually with the prolongation of the treatment time. The mechanical pain sensitivity and thermal allodynia of the PS group were reduced after the operation. The mechanical pain sensitivity and thermal pain sensitivity of the PR group gradually increased with the prolongation of the treatment time, and the 14 days were basically close to the control group. The levels of TNF-*α* and IL-6 in ELISA were significantly higher in the PS group than in the control group, and the content in the PR group was gradually reduced, which was close to the control group. HE staining showed that the sciatic nerve fibers disappeared, and the formation of nerve cavities was obvious in the 14-day PS group. The nerve fibers were found in the sciatic tissue of the PR group, and there was no obvious hemorrhagic edema and cell deformation. The expression of GFAP mRNA in the PS group was significantly higher than that in the control group and the PR group (*p* < 0.05), and the expression of GDNF was opposite (*p* < 0.05). The results of western blot showed that the expression of GFAP protein in the 14-day PS group was significantly higher than that in the control group. The expression of the PR group decreased compared with the control group, and the expression of GDNF was opposite (*p* < 0.05).

**Conclusion:**

Pulsed radiofrequency ablation can promote neurological repair, promote GDNF, and reduce the expression of GFAP in rats with neuropathic pain.

## 1. Introduction

Neuropathic pain (NP) is a common disease that seriously affects the human health and causes impaired mobility. As a fast developing field in neuroscience, NP results from peripheral nerve injury, with such symptoms as heterotopic pain, hyperalgesia, strong burning and tingling sensation, and spontaneous pain in varying degrees [1]. It is an obstacle of daily activities, and the NP secondary to primary injuries induced by transient mechanical damage and to complex cascades triggered by primary injuries will greatly impair the quality of life of the patients. Regarding the complicated pathophysiology of NP, the change in activity of various genes due to the transection of axons can lead to difference in the composition of neurotrophic factors at the injury site, and the sensory axons become the generators of pathological ectopic pulse. The increased density of sodium channel can alter the nerve sensitivity and enlarge the number of membrane receptors in the impaired axons of adrenergic neurons [2]. After the peripheral nerve injury, aberrant structures of sympathetic fibers are formed around the spinal dorsal root ganglion (DRG) neurons, which are regarded as symptoms of sympathetic pain and causes of peripheral nerve injury [3, 4]. In order to reduce the side effects related to the treatment of neural injury, studies have reported that pulsed radiofrequency (PRF), as a kind of nondestructive radiofrequency technology, can treat NP, during which the RF generator produces pulses at a frequency of 2 Hz, with a pause of 5 min, to avoid pathological changes in the tissues at the treatment site [5, 6]. Clinically, pulse repetition frequency has been applied to DRG, brachial plexus, and suprascapular nerve to alleviate the patient's pain, without neural injury-associated side effects [7].

The latest investigation has elaborated that glial fibrillary acidic protein (GFAP), a special marker of astrocytes in the central nervous system, not only supplies nutrition to and promotes regeneration of primary afferent cells but also triggers the sense of pain [8]. A study illustrated that GFAP participates in the mechanism of NP when the dorsal spinal cord of the rats is generated [9]. However, the relationship between astrocytes and NP as well as the pathogeny of NP still remains unclear [10]. Glial cell line-derived neurotrophic factor (GDNF) is an important neurotrophic factor influencing the neuronal survival in peripheral and central nervous system [11]. In addition, researchers have proven that GDNF plays a crucial role in regulating the transmission of pain signals, especially in the NP stage [12]. It exerts its effects on target cells through the receptor complex composed of neural cell adhesion molecules. The intrathecal injection of GDNF into rodents can have a prominent analgesic effect on NP [13, 14], an intractable chronic pain syndrome caused by nervous system injury. GDNF has been found to be able to reverse the changes induced by neural injury, including those of sodium channel expression, neuropeptide, and regulator of G protein signaling 4 [15]. Nevertheless, a study demonstrated that the administration of GDNF to the peripheral tissues will arouse hyperalgesia and inflammatory pain [16]. The receptor components of GDNF are extensively expressed from periphery to spine along the pain pathway. All these studies indicate that the impact of GDNF on pain seemingly depends on the pathological nature and action site [17]. However, no conclusion has been obtained yet. Currently, there has been no report about whether the mechanism of PRF in reducing NP is correlated with the change in GDNF concentration in nerve tissues. Hence, it is essential to elaborate the specific role of GDNF and reveal its mechanism of analgesia.

It was proposed in this research that the effect of PRF on nerve repair can affect the expressions of GFAP and GDNF in NP rats. The classical animal model of NP as well as inflammatory and neurological examinations was utilized, and the variations in the genes and proteins of GFAP and GDNF were examined using quantitative reverse transcription-polymerase chain reaction (qRT-PCR) and Western blotting, so as to uncover the effect of PRF on nerve repair in NP rats and provide an experimental basis and new ideas for developing novel treatments of NP in subsequent studies.

## 2. Materials and Methods

### 2.1. Modeling and Grouping

A total of 30 clean healthy adult Sprague-Dawley (SD) rats were selected and fed at 22-24°C, with humidity of 40-70% and normal circadian rhythm, and they had free access to food and water. Then, all the SD rats were randomly divided into control group (group C), partial sciatic nerve ligation (PSNL) + sham group (group PS), and PSNL + PRF group (group PR). After anesthesia of the rats with 1.5% isoflurane, the skin in the right upper femoral section was cut open under aseptic conditions, the muscles were bluntly dissected to expose the sciatic nerve trunk, and a 7-0 nylon suture was sewn into the nerve trunk to ligate the 1/3-1/2 of the dorsal branch of sciatic nerve. After that, the sciatic nerve was put back to the anatomical position, and the wound was sutured layer by layer till the skin. In group C, only the right sciatic nerve was exposed without ligation. Both the PS group and the PR group used Huang Mincong et al. [18] to establish neurogenic pain rat models in experiments using pSNL surgery. In the PS group, after the pain behavior of the rats became stable, only pulsed radiofrequency localization was performed without pulsed radiofrequency treatment. The rats in group PR were subjected to PSNL and PRF treatment after the pain behaviors were stable. The changes in behavior and other indexes were observed on the 1st, 3rd, 7th, and 14th d of treatment.

### 2.2. PRF Treatment

After successful modeling in group PR, the ligated part of the sciatic nerve was exposed again. Next, a RF pain management system (VATION50M, Sichuan Jinjiang Electronic Science and Technology Co., Ltd.) was employed, the electrical nerve stimulation (0.2 mA) was turned on, and the RF needle was fixed when rhythmic contractions of the right leg occurred. In group PS, only the RF needle was fixed for 4 min, and no PRF was performed. In group PR, 2 cycles of PRF treatment (parameters: 42°C, 2 Hz, 120 s) were conducted for 4 min in total after fixation of the RF needle.

### 2.3. Behavioral Determination

The behaviors of the rats in each group were observed by at least three personnel at the same time point (8 : 00-12 : 00 a.m.) before modeling, at 1, 3, 7, and 14 d after modeling and at 1, 3, 7, and 14 d after PRF in a quiet environment. Finally, the results were summarized.

### 2.4. Determination of Mechanical Hyperalgesia

Von Frey test was adopted to determine the threshold of mechanical hyperalgesia, namely, mechanical withdrawal threshold (MWT). The rats were placed in organic glass cages with a metal lattice mesh at the bottom. Before the test, the rats adapted to the cage environment for 30 min. Later, the skin of foot soles between the third and fourth toes of the hind limb was vertically stimulated using a metal needle of an electronic pain detector through the mesh layer at the bottom of the glass cage, and the stimulus intensity was increased gradually to trigger rapid paw withdrawal and lifting reflexes of the hind limb within about 3 s. Finally, the numerical value of minimum stimulus intensity (g) that produced paw withdrawal reflex was recorded automatically using a recorder, the stimulation was repeated many times, with an interval of 1 min, and the average value was read and recorded.

### 2.5. Determination of Thermal Hyperalgesia

A hot/cold plate analgesia instrument was used to detect the thermalgesia liminal value, namely, thermal withdrawal latency (TWL), of the rats. In a quiet indoor environment at 22°C, the panel temperature of the hot/cold plate analgesia instrument was set as 52°C/s. The instrument was turned on in advance before the test, the rats were put into an organic glass box on the panel when the set temperature (52°C/s) was reached, and the timing button was pressed. When such behavioral intentions as foot stamping, paw licking, and jumping out were observed, the stop button was pressed immediately. After that, the rats were returned to the cages, and the time was recorded. If the rats did not manifest the above behaviors for 20 s, the rats were removed from the glass box promptly to prevent tissue scalding, and the thermalgesia liminal value was recorded as 20 s. Every rat was tested for 5 times, with an interval of 5 min, and the mean value of the middle three values was calculated.

### 2.6. Determination of Inflammatory Factors in Nerve Tissues

Inflammatory factors are vital indexes of neural injury, which can indicate the speed of injury repair, so the content of the inflammatory factors in the sciatic nerve tissues was measured via enzyme-linked immunosorbent assay (ELISA). After the rats were anesthetized by 1.5% isoflurane, the sciatic nerve tissues were separated aseptically, added with strong lysate and broken in a homogenizer, followed by adequate lysis at 4°C, centrifugation at a low temperature and 1,000 g for 10 min, and collection of the supernatant. The changes in the indexes were detected by kits according to the practical situations and specific instructions. Finally, the absorbance of the inflammatory factors in each group was measured using a microplate reader.

### 2.7. Observation of Changes in Sciatic Nerve Tissues via Hematoxylin and Eosin (HE) Staining

At 14 d after operation, the rats were anesthetized by 1.5% isoflurane; the sciatic nerve tissues were isolated under sterile conditions, quickly fixed in tissue fixative for 24 h, and then flushed with running water overnight. Later, the fixed tissues were dehydrated using an automatic dehydrating machine and embedded in paraffin by virtue of an automatic section embedding machine. After deparaffinization, the sections were hydrated in 95%, 90%, 80%, 75%, and 50% ethanol separately, followed by clearing, dipping, and embedding in paraffin. Subsequently, the paraffin-embedded blocks were prepared into about 5 *μ*m-thick pathological sections. Finally, the thin sections were baked dry, stained with hematoxylin for 20 min, separated in hydrochloric acid and ethanol for 30 s, stained with eosin for 12 min, separated in 90% ethanol for 45 s, and mounted and observed under a light microscope.

### 2.8. Detection of Expression of Relevant Genes via RT-PCR

(1) The rats were anesthetized with 1.5% isoflurane to separate the sciatic nerve tissues aseptically, and 100 mg of sterile tissues was carefully and precisely weighed in a low temperature and homogenized using lysis buffer to extract total ribonucleic acid (RNA) in the tissues. After the purity and concentration of RNA were monitored qualified, (2) messenger RNA (mRNA) was reversely transcribed into complementary deoxyribonucleic acid (cDNA), which was stored in a refrigerator at -80°C. (3) The primer amplification was performed using a 20 *μ*L system (2 *μ*L of cDNA, 10 *μ*L of qPCR Mix, 2 *μ*L of primer, and 6 *μ*L of ddH_2_O) for 40 cycles. The primer sequences of target genes and internal reference (glyceraldehyde-3-phosphate dehydrogenase (GAPDH)) were designed based on those on GenBank (Table 1). The expression levels of target genes were detected via qRT-PCR. The relative expression levels of related genes in each group of sciatic nerve tissues were calculated using 2^-△△Ct^ method

### 2.9. Western Blotting Assay

The protein expressions of GFAP and GDNF in each group at 14 d were verified after the aforementioned tests. 200 mg of tissues was weighed into 10 mL EP tubes and then placed on ice. Later, a proper amount of proportionally prepared lysis buffer was added, and the tissues were incubated in the refrigerator to sufficiently lyse the tissues and release the proteins, followed by centrifugation and collection of supernatant. The protein concentration was detected and calculated in accordance with the instructions of BCA kit. After that, Western blotting assay was performed as follows: The proteins were loaded for electrophoresis, transferred onto membranes, and incubated with primary and secondary antibodies. Finally, the images were developed using a gel imaging system, the level of proteins to be detected was corrected via GAPDH, and the grayscale values of the protein bands were analyzed by the ImageLab software.

### 2.10. Statistical Analysis

The data originally recorded in the experiment are processed by the SPSS 22.0 analysis software, and all measurement data are expressed by the mean ± standard deviation (*x* ± SD); the same index was compared at different time points by repeated measures analysis of variance, the differences between groups at each time point were compared by independent samples *t*-test, and statistically significant differences were used *p* < 0.05. At least three replicates for each experiment, the histogram uses GraphPad Prism 7.0.

## 3. Experimental Results

### 3.1. Examination of General Behaviors

Observing the behavioral changes of mice in each group during the first to 14 days of treatment, it was found that the rats in group C could move freely, drink water regularly, and have normal activities, with favorable conditions. Those in group PS manifested different degrees of claudication, weakness of lower extremities, toes put together and everted, neural injury, and other behavioral changes. However, those symptoms were gradually relieved with the prolonged duration of treatment after PRF in group PR, which were basically close to those in group C on the 14th d of treatment.

### 3.2. Mechanical Hyperalgesia (MWT) Determined

As shown in Table 2, the MWT at 1, 3, 7, and 14 d after operation in group PS was remarkably lower than that in group C (*p* < 0.05), while it was notably higher in group PR than that in group PS (*p* < 0.05), approximately equal to that in group C at 14 d.

### 3.3. Thermal Hyperalgesia (TWL) Determined

According to Table 3, group PS had markedly shorter TWL than group C at 1, 3, 7, and 14 d after operation (*p* < 0.05), but group PR had obviously longer TWL than group PS (*p* < 0.05), and the TWL was substantially close to that in group C at 14 d.

### 3.4. Inflammatory Factors in Nerve Tissues Determined

The content of interleukin-1 (IL-1) (Figure 1(a)) and tumor necrosis factor-alpha (TNF-*α*) (Figure 1(b)) was increased at 1, 3, 7, and 14 d after operation in group PS (*p* < 0.05), which was decreased progressively in group PR (*p* < 0.05).

### 3.5. Changes in Sciatic Nerve Tissues Observed via HE Staining

The results of HE staining indicated that the sciatic nerve exhibited no pathological changes but normal structure and orderly arranged nerve cells in group C (Figure 2(a)). The sciatic nerve fibers disappeared, and apparent cavities were formed in group PS (Figure 2(b)). The aggregation of nerve fibers in the sciatic nerve tissues was visible in group PR, without obvious hemorrhage, edema, and cytomorphosis in the tissues (Figure 2(c)).

### 3.6. Expression of Relevant Genes Detected via RT-PCR

The results of RT-PCR assay manifested that GFAP level (Figure 3(a)) was elevated at 1, 3, 7, and 14 d after operation in group PS (*p* < 0.05), while it was lowered in group PR (*p* < 0.05). However, the expression trends of GDNF (Figure 3(b)) were the opposite.

### 3.7. Western Blotting Assay

After the above tests were performed, the protein expressions of GFAP and GDNF in each group were testified at 14 d. It was shown in the protein assay results (Figure 4) that group PS displayed an evidently raised GFAP level at 14 d after operation (*p* < 0.05), while group PR manifested a distinctly reduced GFAP level at 14 d after operation (*p* < 0.05). However, the expression of GDNF manifested the opposite trends.

## 4. Discussion

PRF may be a preferable substitute of traditional RF. According to a prospective randomized clinical study, low-temperature PRF is a safe and efficacious therapeutic method for NP [19]. The heat produced by the pulse can never reach the temperature that destroys the nerves [20]. NP symptoms will not occur when the temperature of PRF stimulus is 42°C [21], thus reducing the risk of reaction of nerve tissues to pain. In this research, PRF was employed to treat NP rats, and it was found through general behavioral observation that the rats in group C exhibited free movement as well as normal drinking and activities in good conditions. Behavioral changes such as claudication, weakness of lower extremities, close and valgus toes, and neural injury in different degrees emerged in group PS. After treatment with PRF in group PR, however, those symptoms were gradually relieved with the prolongation of treatment, which were basically close to those in group C on the 14th d of treatment. The mechanical and thermal hyperalgesia in each group was further observed, and it was discovered that both MWT and TWL declined remarkably at 1, 3, 7, and 14 d after operation in group PS compared with those in group C, while they were notably elevated in group PR in comparison with those in group PS, and the TWL was substantially close to that in group C at 14 d, suggesting that PRF is able to prominently ameliorate the mechanical and thermal hyperalgesia of NP rats. Besides, the results of HE staining indicated that the sciatic nerve exhibited no pathological changes but normal structure and regularly arranged nerve cells in group C. Group PS manifested disappearance of sciatic nerve fibers and formation of obvious cavities. In group PR, the aggregation of nerve fibers was visible in the sciatic nerve tissues, and no significant hemorrhage, edema, and cytomorphosis in the tissues were examined. All those findings are consistent with those in previous studies [22, 23].

The activated DRG neurons can release substance P, which may result in structural change in fibers and rapid development of heterotopic pain [24]. The microglia and astrocytes in the central nervous system can release various proinflammatory cytokines, including PGE2, TNF-*α*, IL-1, and IL-10, which are crucial players in maintaining NP symptoms, further facilitating the occurrence and development of NP [25]. In this research, it was observed that the content of IL-1 and TNF-*α* was increased at 1, 3, 7, and 14 d after operation in group PS, while it was decreased progressively in group PR, which is similar to the results in the studies mentioned above. It was demonstrated in research that the abnormal activation of glial cells can promote NP, and microglia and astrocytes are the major glial cells involved in the process of pain [26]. The activation of glial cells can aggravate the pain, and the immuno-inflammatory responses dominated by neuroglial cells play vital roles in the occurrence and prolongation of NP. GFAP, a specific astrocytic marker, is expressed in the central nervous system. The highly expressed GFAP can damage a variety of central nervous systems [27]. In addition, the regulation of reception, integration, and transmission of NP information is associated with the functions of neurons and astrocytes in the cerebral cortex. A study elaborated that the intrathecal injection of GDNF weakens the expression of GFAP markedly, suggesting that the mechanism of analgesic effect of GDNF has a correlation with the inhibition on astrocytic activation [28]. Based on previous reports, NP-induced activation of astrocytes can be repressed by GDNF through multiple pathways, leading to decreased GFAP expression. GDNF is capable of inhibiting the growth of afferent nerve fibers and the increase in expression of neuropeptide Y that causes NP. It can also stimulate the release of endogenous analgesic substances such as somatostatin [29]. In this research, the PCR assay revealed that the level of GFAP was elevated, while GDNF level was lowered in group PS at 1, 3, 7, and 14 d after operation. However, group PR had a reduced GFAP level and a raised GDNF level at 1, 3, 7, and 14 d after operation. The same changes were observed in the protein assay, elucidating that PRF can suppress GFAP expression by activating the expression of GDNF, thereby exerting a restorative effect on NP. Such changes were confirmed in this research, and the effects of PRF on nerve repair and expressions of GFAP and GDNF in NP rats can be further explored using in vitro culture of cell lines and numerous molecular biological methods in the future.

In conclusion, NP will trigger a series of pathological changes such as inflammatory responses and neurological dysfunction, while PRF can prominently inhibit the incidence of NP and the expression of GFAP by activating GDNF expression, thus restoring NP. The more detailed effects can be investigated later using more molecular means. In a word, this study provides theoretical bases for the prevention and treatment of NP as well as new ideas and experimental bases for subsequent in-depth studies.

## Figures and Tables

**Figure 1:** Content of inflammatory factors: (a) the content of IL-1; (b) the content of TNF-*α*. The content of IL-1 and TNF-*α* is increased at 1, 3, 7, and 14 d after operation in group PS (*p* < 0.05), which is decreased progressively in group PR (*p* < 0.05). ^a^*p* < 0.05 vs. group C; ^b^*p* < 0.05 vs. group PS.

**Figure 2:** HE staining. (a) The sciatic nerve exhibits no pathological changes but normal structure and orderly arranged nerve cells in group C. (b) The sciatic nerve fibers disappear, and apparent cavities are formed in group PS. (c) The aggregation of nerve fibers in the sciatic nerve tissues is visible in group PR, without obvious hemorrhage, edema, and cytomorphosis in the tissues.

**Figure 3:** RT-PCR assay results: (a) expression level of GFAP; (b) expression level of GDNF. GFAP level is elevated at 1, 3, 7, and 14 d after operation in group PS (*p* < 0.05), while it is lowered in group PR (*p* < 0.05), and the expression trends of GDNF are the opposite. ^a^*p* < 0.05 vs. group C; ^b^*p* < 0.05 vs. group PS.

**Figure 4:** Results of protein assay. Group PS displays an evidently raised GFAP level at 14 d after operation (*p* < 0.05), while group PR manifests a distinctly reduced GFAP level at 14 d after operation (*p* < 0.05). However, the expression of GDNF manifests the opposite trends. ^a^*p* < 0.05 vs. group C; ^b^*p* < 0.05 vs. group PS.

**Table 1:** Primer sequences.

Target gene	Primer sequence (F-R)
GAPDH	5′-GATGGTGGGTATGGTCAGAAGGA-3′ 5′-GCTCATTGCCGATAGTGATGACCT-3′
GDNF	5′-ATGAAGTTATGGGATGTCGT-3′ 5′-CAGGGTCAGATACATCCACA-3′
GFAP	5′-GGACTCCCTGAAGACCAATATGGAAG-3′ 5′-GCATTGAGCTAGATGGGTTAATGTTG-3′

**Table 2:** Results of MWT determined (g).

Group	Before operation	1 d after operation	3 d after operation	7 d after operation	14 d after operation
Group C	16.3 ± 0.8	16.3 ± 0.8	16.3 ± 0.8	16.3 ± 0.8	16.3 ± 0.8
Group PS	16.1 ± 0.9	10.5 ± 0.2^a^	8.1 ± 0.7^a^	6.5 ± 0.6^a^	3.7 ± 0.4^a^
Group PR	16.2 ± 0.7	14.6 ± 0.3^b^	13.5 ± 0.4^b^	12 ± 0.7^b^	15.9 ± 0.8^b^

Results of MWT determined. The MWT at 1, 3, 7, and 14 d after operation in group PS is remarkably lower than that in group C (*p* < 0.05), while it is notably higher in group PR than that in group PS before operation and at 1, 3, 7, and 14 d after operation (*p* < 0.05). ^a^*p* < 0.05 vs. group C; ^b^*p* < 0.05 vs. group PS.

**Table 3:** Results of TWL determined (Sec).

Group	Before operation	1 d after operation	3 d after operation	7 d after operation	14 d after operation
Group C	1.83 ± 0.23	1.82 ± 0.21	1.83 ± 0.20	1.82 ± 0.20	1.80 ± 0.29
Group PS	1.81 ± 0.18	1.4 ± 0.12^a^	1.2 ± 0.13^a^	0.8 ± 0.18^a^	0.5 ± 0.21^a^
Group PR	1.82 ± 0.09	1.68 ± 0.14^b^	1.49 ± 0.10^b^	1.25 ± 0.21^b^	1.79 ± 0.32^b^

Results of TWL determined. Group PS has markedly shorter TWL than group C at 1, 3, 7, and 14 d after operation (*p* < 0.05), but group PR has obviously longer TWL than group PS (*p* < 0.05). ^a^*p* < 0.05 vs. group C; ^b^*p* < 0.05 vs. group PS.

## Data Availability

The datasets used and/or analyzed during the current study are available from the corresponding author on reasonable request.
